RETRACTED

# Bayesian‐Edge system for classification and segmentation of skin lesions in Internet of Medical Things

**DOI:** 10.1111/srt.13878

**Published:** 2024-07-31

**Authors:** Shahid Naseem, Muhammad Anwar, Muhammad Faheem, Muhammad Fayyaz, Muhammad Sheraz Arshad Malik

**Affiliations:** ^1^ Department of Information Sciences Division of Science and Technology University of Education Lahore Pakistan; ^2^ School of Technology and Innovations University of Vaasa Vaasa Finland; ^3^ Department of Computer Science FAST National University of Computer & Emerging Sciences Chiniot‐Faisalabad Campus Islamabad Pakistan; ^4^ Department of Software Engineering Government College University Faisalabad Faisalabad Pakistan

**Keywords:** auto‐immune pathogenic traits, Bayesian inference, edge intelligence, internet of things, malignance, psoriasis, skin lesions

## Abstract

**Background:**

Skin diseases are severe diseases. Identification of these severe diseases depends upon the abstraction of atypical skin regions. The segmentation of these skin diseases is essential to rheumatologists in risk impost and for valuable and vital decision‐making. Skin lesion segmentation from images is a crucial step toward achieving this goal—timely exposure of malignancy in psoriasis expressively intensifies the persistence ratio. Defies occur when people presume skin diseases they have without accurately and precisely incepted. However, analyzing malignancy at runtime is a big challenge due to the truncated distinction of the visual similarity between malignance and non‐malignance lesions. However, images' different shapes, contrast, and vibrations make skin lesion segmentation challenging. Recently, various researchers have explored the applicability of deep learning models to skin lesion segmentation.

**Materials and methods:**

This paper introduces a skin lesions segmentation model that integrates two intelligent methodologies: Bayesian inference and edge intelligence. In the segmentation model, we deal with edge intelligence to utilize the texture features for the segmentation of skin lesions. In contrast, Bayesian inference enhances skin lesion segmentation's accuracy and efficiency.

**Results:**

We analyze our work along several dimensions, including input data (datasets, preprocessing, and synthetic data generation), model design (architecture, modules), and evaluation aspects (data annotation requirements and segmentation performance). We discuss these dimensions from seminal works and a systematic viewpoint and examine how these dimensions have influenced current trends.

**Conclusion:**

We summarize our work with previously used techniques in a comprehensive table to facilitate comparisons. Our experimental results show that Bayesian‐Edge networks can boost the diagnostic performance of skin lesions by up to 87.80% without incurring additional parameters of heavy computation.

RETRACTED

## 1 INTRODUCTION

Skin is a prime structure of the human body and is directly exposed to air, leading to most skin diseases and illnesses. It might occur in any culture, at any stage in human life, and affect almost 30% to 70% or even more people. Skin lesion detection and segmentation are also useful as preprocessing steps when analyzing wide‐field images with multiple lesions.^1^ However, despite the importance of lesion segmentation, manual delineation of skin lesions remains a laborious task that suffers from significant inter‐ and intra‐observer variability. Consequently, a fast, reliable, and automated segmentation algorithm is needed. There are two main types of skin lesions: primary lesions (e.g., Macule, Patch, Papule, Plaque, Vesicle, Bulla, Pustule, and Nodule), whereas secondary lesions (e.g., Atrophy, Scaling, Crust, Tylosis, and Excoriation). Its early diagnosis is critical for a good prognosis: melanoma can be cured with a simple outpatient surgery if detected early, but the 5‐year survival rate drops from over 99% to 30% if it is diagnosed at advanced stages. These two modalities are commonly employed in automated skin lesion analysis.

### 1.1 Classification and segmentation of skin lesions

Segmentation is the partitioning of an image into meaningful regions. Semantic segmentation, in particular, assigns appropriate class labels to each area. The task is usually binary for skin lesions, separating the lesion from the surrounding skin. Illumination and contrast issues, intrinsic interclass similarities and intra‐class variability, occlusions, artifacts, and the diversity of imaging tools hinder automated skin lesion segmentation. The lack of large datasets with ground‐trust segmentation masks generated by experts compounds the problem, impeding the training of models and their reliable evaluation. Natural artifacts such as blood vessels and artificial ones such as surgical marker annotations and Len artifacts (dark corners occlude skin lesion images. Intrinsic factors such as lesion size and shape variations, different skin colors, low contrast, and ambiguous boundaries complicate the automated segmentation of skin lesions.^2^

Segmentation is a challenging and critical operation in the automated skin lesion analysis workflow. Rule‐based skin lesion diagnostic systems, popular in the clinical setting, rely on an accurate lesion segmentation to estimate diagnostic criteria such as asymmetry, border irregularity, and lesion size, as needed for implementing the edge intelligence algorithm. By contrast, in deep learning (DL)‐based diagnostic systems, restricting the areas within an image, thereby focusing the model on the lesions' interior, can improve classification robustness. For example, recent studies have shown the utility of segmentation in improving the deep‐learning‐based classification performance for specific diagnostic categories by regularizing attention maps, allowing the cropping of lesion images, tracking lesions' evolution, and removing imaging artifacts. In the Edge Learning (EL)‐based skin lesion classification and segmentation framework, presenting the delineated skin lesion to the user can also help interpret the DL black box. Thus, it may instill trust or raise suspicion about the Bayesian Inference Segmentation (BIS) for skin lesions.^3^

RETRACTED

### 1.2 Edge intelligence

Artificial intelligence has made rapid progress in image recognition over the last decade, using machine learning (ML) and DL methods. Segmentation and classification models can be developed using traditional ML and DL methods. Traditional ML methods have more superficial structures than DL methods, which use extracted and selected features as input.^4^ The DL method can automatically discover underlying patterns and identify the most descriptive and salient features in image recognition and processing tasks. The progress has significantly motivated medical workers to explore the potential for applying AI methods in disease diagnosis, particularly skin disease diagnosis.^5^ DL approaches can learn hierarchical features and extract high‐level and influential characteristics from images. Both supervised and unsupervised DL approaches are used for effective computational segmentation. Edge‐based segmentation methods, such as the watershed algorithm, utilize intensity changes among adjacent pixels to outline the boundary of a skin lesion. The process is susceptible to noise, such as skin texture and air bubbles, which can lead to convergence, especially around noisy points, and produce erroneous segmentation results.^6^ The edge intelligence segmentation method often needs help to achieve accuracy when segmenting images with noise, low contrast, and varied color and texture.^9^ After studying different literature about psoriasis, it was observed that mostly men, women, and adults between the ages of 15 and 25 are infected with this disease. Timely exposure to malignancy in psoriasis can update the persistence ratio of skin‐infected patients. However, the manual detection of malignancy requires massive requests for specialists and agonizes from interobserver divergences.^7^ Most research has been based on biological therapies for skin disease patients for the last few years. Rather than having some side effects on skin disease patients, these biological therapies provide a selective and immunologically direct intervention to the patients.^8^ Although most common techniques and technologies, including a biochemical and immune system, that is, used for diagnosing skin diseases, are more accurate and efficient for visual inspection and auscultation, visual inspection through the naked eye is considered to be an effective way to acquire authenticated information about the skin affected persons including their distribution form, skin color and shape of the affected area and firm auscultation.^9^ Primary skin lesions shown in Figure 1 include macules, patches, papules, plaques, vesicles, bulla, pustules, and nodules. These lesions occur as an unswerving effect of the disease process. Most of these diseases are temporarily evaluated.

RETRACTED

**FIGURE 1:** Primary skin lesions contain primary skin lesions such as macules, patches, papules, plaques, vesicles, bulla, pustules, and nodules that occur as an unswerving effect of the disease process.

Figure 2 shows that patients modify Secondary lesions because of rubbing, scratching, local applications, or treatment. They are not path gnomic of any particular disease.

**FIGURE 2:** Secondary skin lesions are because by rubbing, scratching, local applications, or treatment such as atrophy, scaling, crust, Tylosis, and excoriation.

### 1.3 Structure of the research paper

Section 1 includes an introduction, classification, and segmentation of skin lesions and edge intelligence. Section 2 consists of the literature review. Section 3 includes related work and a Bayesian‐Edge Model for skin lesion detection, classification, and segmentation. Section 4 includes experimental results. Section 5 includes results and discussion. Section 6 concludes the research article and provides some future suggestions to help researchers contribute to future research.

## 2 LITERATURE REVIEW

In their work, Armstrong^10^ delved into the intricacies of psoriasis, describing it as a persistent condition that can affect human skin, presenting as red patches that may appear anywhere on the body, such as the knees, elbows, and lips. Psoriasis is a chronic inflammatory skin disorder with a substantial genetic inclination and autoimmune pathogenic characteristics, making it a complex and multifaceted disease. These patches, which can vary in size and location, frequently emerge on the elbows, knees, and scalp. In a study by Whan et al.,^11^ it was highlighted that approximately 90% of psoriasis cases are attributed to the chronic plaque‐type variant. This form is characterized by distinct, reddened, itchy plaques covered in silver‐colored scales. These plaques have the potential to merge and cover sizable skin areas, commonly affecting the trunk, the extended surfaces of the limbs, and the scalp. Exploring this topic further,Vincenzo^12^ delved into that psoriasis primarily impacts the skin but can also involve the joints and has links to various other medical conditions. Inflammation extends beyond the psoriasis skin and affects dermatological aspects and other health domains. Compared to individuals without psoriasis, those with the condition display heightened instances of hyperglycemia, hypertension, coronary artery disease, and an elevated body mass index. Notably, the metabolic syndrome, encompassing these conditions above within a single individual, was observed to be twice as prevalent among psoriasis patients. In the study conducted by Gorman et al.,^13^ the authors addressed the prevailing method for diagnosing common skin conditions, which predominantly relies on visual observation. Medical professionals formulate their assessments and recommend treatments based on visual cues and established empirical criteria during the diagnostic process. However, many skin ailments necessitate comprehensive analysis and sometimes involve procedures like biopsies to ascertain their underlying causes accurately. In the context of determining the precise cause of these skin issues,Rendon^14^ pointed out that dermatologists rely on their accumulated expertise to analyze the information gleaned from skin lesions and incorporate empirical guidelines to make a diagnosis. Nevertheless, it is important to note that diagnosing skin lesions solely through observation remains contingent upon the extensive experience of dermatologists. In a separate research effort by Zeeshan et al.,^15^ a framework for categorizing skin images was established, encompassing a variety of image types, including epidemiologic and pigmented variations. It was highlighted that skin conditions can lead to various other diseases, including cancer and paralysis. Nonetheless, practical approaches are available to diagnose and address these conditions at their earliest stages.

RETRACTED

Gerdes et al's publication^16^ elucidated that psoriasis is a persistent inflammatory ailment characterized by manifestations encompassing red, scaly, itchy, and sometimes painful patches, plaques, or bumps. These symptoms typically exhibit a preference for manifesting on the scalp and extensor surfaces of the body, although they can become widespread in severe instances. Remarkably, around 40% of individuals with psoriasis eventually develop psoriatic arthritis, often within 5 to 10 years of psoriasis onset. They are exploring the prevalence of psoriasis; a study by Daragahr et al.^17^ documented variations in its occurrence across different regions globally. Notably, countries with a predominantly Caucasian population frequently record a prevalence ranging from 1% to 3%. The onset of the disease follows a bimodal pattern, with one peak occurring between 15 and 20 years of age. An innovative approach to computer‐aided classification was introduced in a separate investigation by Holmes et al.^18^ This method involved extracting relevant features from various skin attributes using a neural network approach, followed by classifying these features using a support vector machine. The researchers acknowledged, however, that their proposed system has certain limitations, particularly in encompassing a wide range of skin diseases.

The study by Mease and Armstrong ^19^ discussed the complexity of segmenting multi‐disease classifications owing to the diverse characteristics and varying locations of these conditions on the human body. Malignant melanoma and benign lesions, known for their distinct shapes and well‐defined boundaries, permit the relatively straightforward extraction of shape and geometric features from them. Another study by Irmina^20^ underscored the crucial role of color features in multi‐disease classification. Color features were identified as vital in differentiating between various skin diseases. Addressing the healthcare divide between rural and urban areas ^21^ Hammed et al. emphasized the significance of usability indicators in a web portal within a telehealthcare program. They collected data from urban and rural locations across different countries, revealing that urban patients exhibited higher engagement with the web portal, accessing more advanced information. This highlighted the service disparity in rural regions and the imperative to develop enhanced services. An innovative IoT‐based protocol designed by  Seth et al.^22^ aimed to remotely monitor skin lesion data and provide care to elderly individuals at home. This protocol is anticipated to be cost‐effective, improve the quality of life, offer real‐time analysis and categorization, and contribute to the early detection and diagnosis of skin conditions. It is seen as a potential solution for addressing challenges people face in remote areas, where access to adequate skin care facilities is limited.

In a skin tumor screening context by Hameed et al.,^23^ the diagnostic accuracy of clinical dermoscopic image tele‐evaluation was evaluated. Using images collected over time via a mobile phone camera, they demonstrated that clinical image tele‐evaluation could be a viable method for mobile tumor screening.,Chen^24^ outlined diverse systems for classifying and categorizing skin lesions, focusing on pattern classification of dermoscopic images within a perceptually uniform model. Various techniques for lesion segmentation were defined by Rashid,^25^ including clustering, edge‐based, region‐based, and active contour methods. Active contours were highlighted as a commonly used approach. Intelligent edge contour methods were popular for image feature extraction, particularly within the edge intelligence methodology, which uses image intensity to group pixels. A study by Vesal^30^ introduced an edge model dependent on the investigation of curvelet coefficients. The results demonstrated an increase in decomposition scale‐based edges. This approach aimed to aid individuals in conducting self‐examinations for skin diseases.

RETRACTED

Vesal proposed a supervised method called SkinNet, a modified version of U‐Net for the segmentation of skin lesions that contains a more significant number of images from seborrheic keratosis, benign nevus, melanoma, etc. by Kroemer et al.^26^ Al‐Masni proposed a full‐resolution convolutional network for skin lesion segmentation. This method can directly learn the full‐resolution features of each pixel of the input data without preprocessing. The segmentation of skin lesions with find boundaries was reported compared with the results from other DL approaches, such as the fully convolutional network, U‐Net, and SegNet, under the same conditions and with the same datasets.^27^

According to Situ,^28^ pigmented skin lesions (PSLs) can be medically and esthetically problematic, with melanoma being the most concerning form as it is a type of skin cancer. In the United States, it is estimated that one in five Americans will develop skin cancer by age 70, and more than two people die every hour from this condition. Having frequent sunburn increases the risk of developing melanoma. Although the number of newly diagnosed cases is predicted to decrease by 2023, the number of deaths from melanoma is expected to rise. However, early detection significantly increases the 5‐year survival rate for melanoma, which currently stands at 99%.  Dermoscopic images and biopsy images are commonly used to examine PSLs. Dermoscopic images are preferred as they are noninvasive, quick, and cost‐effective. However, there are challenges in accurately interpreting these images, such as the presence of artifacts, variability within and between image classes, and subjective reading by doctors.

The study in Dijimeli^29^ predicts a 15‐year progression of clinical signs of African skin aging, considering endogenous and exogenous factors and developing Causal Bayesian Belief Networks (CBBNs) using expert knowledge from dermatologists. For forehead wrinkles, the evaluation model has been detailed. Specific atlas and extrinsic factors of facial aging were used for this skin type. The prediction method has been validated for all prototypes and all clinical signs of facial aging. CBBNs represent the causal relationships between risk factors and their influence on skin aging progression. They provide a framework for assessing the impact of various lifestyle habits. Their intuitive representation, made of nodes and arcs, makes them both user‐friendly and easy to interpret.  The robust CBBNs formed the mathematical backbone of this expert‐driven modeling, facilitating the simulation of aging trajectories.

RETRACTED

Vesal et al. in their study^30^ introduced a new algorithm, SharpRazor, to detect hair and ruler marks and remove them from the image. The Sharprazor techniques promise to remove and paint dark and white hair in various lesions.  This multiple‐filter approach detects hairs of varying widths within varying backgrounds while avoiding the detection of vessels and bubbles. This algorithm utilizes grayscale plane modification, hair enhancement, segmentation using tri‐directional gradients, and multiple filters for hair varying widths. They developed an alternate entropy‐based processing adaptive thresholding method. White or light‐colored hair and ruler marks are detected separately and added to the final hair mask. A classifier removes noise objects. Finally, a new technique of inpainting is presented, and this is utilized to remove the detected object from the lesion image. It consists of seven main steps: (1) The red color plane image is transformed by smoothing and linear scaling. (2) Two‐directional filters enhance hair images. (3) Gradients in three directions are used to detect maximum hair edges. (4) The image is binarized using an adaptive threshold. (5) White or light‐colored hairs and ruler marks, overlooked in other studies, are detected and combined with the hair mask. (6) Finally, a random forest classifier identifies and removes non‐hair objects. (7) Using the hair mask as a guide, a novel inpainting method removes the detected regions for the original image. 

Al‐Masni et al. in their study^31^ used hybrid DL techniques to segment and classify skin lesions from dermoscopy images—Mask Region‐based Convolutional Neural Network (MRCNN) for semantic segmentation and ResNet50 for lesion detection. The MRCNN is used to pinpoint the precise location of a skin lesion for border delineation. ResNet can learn complex properties and patterns from data to its use of skin connections and residual blocks. Images of skin lesions exhibit advanced ResNet features. ResNet powers the combination of ResNet and MRCNN. The proposed method for classifying skin lesions can be broken down into several phases. First, photos are taken from IoMT gadgets, or an image database is created for classifier training. They amass a huge, annotated collection of dermoscopy images for thorough model training. Using this dataset, the hybrid DL model is trained to capture subtle representations of the pictures from start to finish. Initially, they developed different thresholding techniques for improving record images, eliminating hairs and other artifacts, or enhancing understanding of skin lesions.  Second, skin lesion classification is aided by locating and segmenting the lesions. Last, ResNet can train deep networks without causing the gradients to evaporate or become artificially inflated. These characteristics are used by the MRCNN's central instances segmentation and bounding box regression. The head of MRCNN tweaks ResNet features maps to focus on areas with lesions. To improve classification precision, MRCNN segmentation masks provide damage at the pixel level. The results of MRCNN and ResNET can be used to categorize skin lesions. 

RETRACTED

## 3 PROPOSED SCHEME

In this research, we have proposed a Bayesian‐Edge Model that uses an approximate Bayesian inference to output an uncertainty estimate and its prediction in skin lesion classification and segmentation. The proposed framework is general enough to support various medical machine‐learning tasks and applications. Our results demonstrate the confidence ratings' effectiveness in improving the medical experts' diagnosis performance and reducing the physician workload. In this model, we formulate metrics to evaluate the uncertainty estimation performance of the Bayesian Edge system. These metrics provide an informative tool to compare the quality of uncertainty estimations obtained from various models. Moreover, it hints at choosing an appropriate uncertainty threshold to reject samples and refer them to the physician for further inspection. We provide an in‐depth analysis of skin lesion metrics via the Bayesian‐Edge system to improve team diagnosis accuracy.^32^

A Bayesian edge is the probabilistic version of the artificial neural network, which places a prior distribution over the network's parameter and outputs a probability distribution over the system's parameters that expresses our belief regarding how likely the different model's parameter values are. Therefore, given a new test sample, a Bayesian edge outputs a predictive posterior distribution over class membership probabilities by integrating over the posterior. Moreover, the dispersion of this predictive posterior reflects the reliability of the prediction, yielding the model's uncertainty to its predictions.  In the Bayesian edge system, predicting the unknown label is equivalent to using an ensemble of various configurations of the weights. Therefore, much effort has been put into approximating Bayesian‐Edge systems to make them easier to train. However, some of the approximation methods do not scale to very large datasets.^33^

RETRACTED

This comprehensive dataset is harmonized after aggregation from various sources. Addressing the concern of data imbalance during model training is pivotal, as an imbalanced dataset could bias the model toward the more represented class. To mitigate this, a stratified sampling technique is adopted to create a balanced dataset. The dataset retrieved from the sources above is methodically categorized based on disease attributes, and subsequent random down‐sampling is employed. Given that the Psoriasis category contains a limited number of images (*N* = 1500), other categories in the dataset are down‐sampled to achieve equilibrium. Following the down‐sampling process, 1600 images sized 227 × 227 × 3 are utilized for training and testing the classification model. The precise breakdown of dataset partitioning used in the study is presented in detail in Table 1 and Figure 3.

**TABLE 1:** Different lesion categories.

Sr. no.	Lesions category	No. of images
1.	Plaque	300
2.	Guttate	300
3.	Scalp	300
4.	Pustular	300
5.	Erythrodermic	300
	Total	1500

**FIGURE 3:** Shows different numbers of skin lesions including plaque, guttate, scalp, pustular, erythrodermic, etc.

### 3.1 Bayesian‐Edge model for skin lesion detection

The border or edge detection process within an image yields crucial and clarified insights about its content. Effective edge detection holds the potential to enhance image classification outcomes significantly. This research paper introduces an algorithm tailored for the segmentation and classification of skin images to assess the erythema and scariness of skin lesions. The proposed algorithm classifies diverse skin disease images by utilizing probability values. It combines segmentation and classification techniques to categorize incoming skin disease images. The approach's core involves extracting a discerning array of features from skin lesions, which optimizes subsequent classification processes. After feature extraction, an edge intelligence algorithm can be trained to classify test samples into known categories. Detecting the edges of skin lesions is pivotal in constructing an automated diagnostic system. However, the intricate nature of skin lesions and the complexities of human physiology make precise edge detection particularly challenging. In skin lesions, edge detection is carried out concurrently during segmentation.^34^

RETRACTED

### 3.2 Bayesian‐Edge model for classification and segmentation of skin lesions

An image's border or edge detection processes yield crucial and clarified insights about its content. Effective edge detection holds the potential to enhance image classification outcomes significantly. This research paper introduces an algorithm tailored for the segmentation and classification of skin images to assess the erythema and scariness of skin lesions. The proposed algorithm classifies diverse skin disease images by utilizing probability values. It combines segmentation and classification techniques to categorize incoming skin disease images. The approach's core involves extracting a discerning array of features from skin lesions, which optimizes subsequent classification processes. After feature extraction, an edge intelligence algorithm can be trained to classify test samples into known categories. Detecting the edges of skin lesions is pivotal in constructing an automated diagnostic system. A proficient diagnostic system ensures accurate identification and detection of skin lesion conditions, facilitating the creation of an effective automated skin lesion segmentation tool. Numerous edge detection methods have been presented in the literature for various applications. However, the intricate nature of skin lesions and the complexities of human physiology make precise edge detection particularly challenging. In skin lesions, edge detection is carried out concurrently during segmentation.^35^

Figure 4 illustrates edge intelligence, a segmentation methodology rooted in image processing, for detecting skin lesions within human skin images. The main objectives of this research are as below:

1. To identify the commonly available datasets that could be accessed freely.
2. To explore the contribution and limitations of the current state‐of‐the‐art methods.
3. To present the summary of the open challenges in skin disease and cancer detection and classification. To increase the accuracy of skin disease detection. Three essential features in image classification are texture, color, shape, and a combination of these diseases.
4. To identify the edges of objects within skin disease images or segment the image into regions of interest and nonrelevant areas.
5. Accurate image detection and segmentation are prerequisites for effective and efficient computer‐aided systems.

**FIGURE 4:** Bayesian‐Edge intelligence‐based skin lesions segregation image processing, for the detection of skin lesions within human skin images.

RETRACTED

The final image output is generated using an artificial intelligence technique called ant colony optimization. A three‐stage preprocessing approach is initially employed to refine the quality of skin lesion images. This involves color space conversion, contrast enhancement, and filtering, all of which contribute to elevating the overall quality of the skin lesion image. This figure defines the procedure for extracting the psoriasis images attributed to the edge intelligence technique. Using this method, we first locate the skin lesions on the infected skin and then measure the image's features as indicated in Equations ((1), (2), (3), (4)).

(1) $$\mu \;=\sum_{i=0}P\left(i\right)$$

(2) $$\sigma^{2}=\sum_{i=0}^{G-1}{\left(i-u\right)}^{2}\left(i\right)$$

(3) $$E\;=\sum_{i=0}^{G-1}{\left(i\right)}^{2}$$

(4) $$H\;=\sum_{i=0}^{G-1}\left(i\right)\mathrm{lo}g_{2}\left[p\left(i\right)\right]$$

where

μ=Meanvaluetolocatetheskinlesionsoninfectedskin,

$\;\sigma^{2}=MediancalculatedfromMeanvaluesofinfectedskin\left(i\right)$,

 H=Estimatedtheinfectedfeaturesclassification.

These formulae evaluate the skin lesions of infected skin values. These values indicate whether a person's skin is healthy or unhealthy. If diseases are present in the input photos, the numerical parameter identifies and separates them. Define a two space variables function f(*x,y*) of two space variables x and y, where *x* = 0,1, etc., to calculate the mathematical parameter of an image in this.N‐1 and *y* = 0,1,………M‐1. Function f(*x*,*y*) can have discrete values with *i* = 0,1,…G, where G is the overall image intensity level. The function that displays the number of pixels in the entire image is the intensity level histogram Invalid source specified.

Bayesian inference with a parameter set contains optimal segregation rules under the maximum likelihood (ML) to classify an observed feature vector of dimensions to one of the class labels. The skin lesions of infected skin values are evaluated by these formulae. These values indicate whether a person's skin is healthy or unhealthy. If diseases are present in the input photos, the numerical parameter identifies and separates them. Define a two space variables function f(*x,y*) of two space variables x and y, where *x* = 0,1, etc., to calculate the mathematical parameter of an image in this.N‐1 and *y* = 0,1,………M‐1. Function f(x,y) can have discrete values with *i* = 0,1,…G, where G is the overall image intensity level. The function that displays the number of pixels in the entire image is the intensity level histogram Invalid source specified.  Bayesian inference with a parameter set contains optimal segregation rules under the maximum likelihood (ML) to classify an observed feature vector of dimensions to one of the class labels, which is given in Equation (5):

(5) $$\hat{C}=\arg_{c}^{\max}P\left(X|c;\theta \right)$$

where

$\hat{C\;}=Bayesian\;inference,$ $\arg_{c}^{\max}P=Maximum\;Likelyhood\;estimators$,

X=numberofinputimages,

C=Imageclasslabels.

RETRACTED

Bayesian inference employs two distinct approaches for data classification. The first approach focuses on selecting the network structure, thereby establishing relationships among variables. Meanwhile, the second approach centers on defining feature distributions. These features can manifest as discrete entities whose distributions adopt probability mass functions. Conversely, selecting a distribution is imperative if the features are continuous, with the Gaussian distribution being the most prevalent choice. A specific subset within Bayesian inference is the Naive Bayes (NB) classifier. The foundation of the NB classifier lies in assuming that, given the class label, all features are conditionally independent. Although this assumption often deviates from reality, NB has demonstrated successful implementation across numerous classification scenarios. The efficiency of NB is attributed to its demand for a relatively small number of parameters that require learning. If the features X are assumed to be independent of each other conditioned upon the class label c, Equation (6) reduces to:

(6) $$\hat{c}=\arg\max\prod P\left(X|c;\theta \right)$$

Identifying a maximum weighted spanning tree entails determining a collection of arcs that link features in a manner where the resultant graph forms a tree structure, and the combined weights of these arcs are maximized. In the context of the expanding array of applications and algorithms that effectively utilize unlabeled data, combined with the emergence of theoretical considerations surrounding the efficacy of unlabeled data in specific scenarios, the concept of semi‐supervised learning gains prominence. This learning paradigm is regarded with optimism, as it can alleviate the burden on practitioners by reducing the necessity for amassing extensive sets of costly labeled training data.

A pair of values (c, x) is derived from the distribution P(C, X). Subsequently, the value of c can be revealed, or the sample may remain devoid of a label. The constant probability of a labeled sample, denoted as λ, remains fixed and independent of the samples. When working with the same underlying distribution P(C, X) to model samples, with some samples treated as unlabeled, the estimation of θ ^ is conducted using maximum likelihood. The distribution P(C, X|θ) can be decomposed in two ways: either as P(C, X|θ) P(X|θ) or as P(X|C, θ) P(X|θ). The log‐likelihood function for this model, considering a dataset comprising both labeled and unlabeled data, can be expressed in Equation ((7), (8), (9)):

(7) $$L\;\left(\theta \right)=L_{i}\;\left(\theta \right)+\log\left(\lambda^{N_{i}}{\left(1-\lambda \right)}^{N_{u}}\right.$$

(8) $$L_{i}\;\left(\theta \right)=\sum_{i=1}^{N_{i}}\log\left[\underset{c}{∐}\left(p\left(C=c^{/}|\theta \right)p\left(X_{j}|c^{/},\theta \right)I_{{\left\{C=c^{/}\right\}}^{\left(c_{i}\right)}}\right.\right]$$

(9)

where

$c_{i}\;\left(x\right)=derived\;values$ $\;x_{i}=random\;sample$ P(C,X)=distributedvalues c=Sampleofskininfecteddata θ=estimatedconductedusingmaximumlikelihood λ=labeleddata $P(C=c^{⋰})=MaximumCoefficient$ L=Likelihoodfunction $\;N_{i}=Prior\;data$ $\;N_{\mu }=Mean\;data$

The mixing coefficients are denoted as P(C = c^/^). Leveraging the indicator function offers a conventional approach to compute probabilities through the assessment of expected values. To illustrate, the efficacy of Bayesian inference hinges on the accurate segregation of skin lesions. In the Bayesian‐Edge model, if high model uncertainty is indicative of erroneous predictions, it can be leveraged to mimic the clinical workflow and select proper subsets of the samples with uncertain diagnoses for further testing by an expert. This procedure will eventually increase the prediction performance of the automated system, thus building the experts’ trust in such systems. More specifically, we want the final automated systems to detect skin lesions. If the Bayesian‐Edge model predicts the skin lesions sample correctly, it does not necessarily require to be certain on the same sample. If the proposed model, for instance, correctly detects a skin sample, but with relatively higher uncertainty. This can happen if the sample is rarely presented to the model in such a pose or condition. It can be summarized in Equation (10), (11), ^36^:

(10) $$P_{\mathrm{Hr}}\;\left(\mathrm{correct}|\mathrm{certain}\right)=\frac{P\left(\mathrm{correct},\mathrm{certain}\right)}{P\left(\mathrm{certain}\right)}=\frac{N_{\mathrm{cc}}}{N_{\mathrm{cc}}+N_{\mathrm{ic}}}$$

(11) $$\begin{array}{ccc} P_{\mathrm{Hr}}\;\left(\mathrm{uncertain}|\mathrm{incorrect}\right) & = & \frac{P\left(\mathrm{uncertain},\mathrm{incorrect}\right)}{P\left(\mathrm{incorrect}\right)}=\frac{N_{\mathrm{iu}}}{N_{\mathrm{iu}}+N_{\mathrm{ic}}}\\ & = & R_{\mathrm{iu}}\left(\mathrm{HT}\right) \end{array}$$

where N and R represent the count and ratio for each combination, we can also measure the overall accuracy of the uncertainty estimation as the ratio of the desired cases (i.e., correct–certain and incorrect–uncertain) over all possible cases.

RETRACTED

### 3.3 Data description

We used the publicly available HAM 10 000 dataset of skin lesion samples to evaluate the Bayesian‐Edge system's accuracy for skin lesion diagnostics. This dataset contains dermoscopic images of the most important diagnostic categories in the realm of pigmented lesions collected from a diverse population and different modalities. Expert pathologies label images as one of the seven categories of Melanoma, as shown in Figure 5.

**FIGURE 5:** Illustrating skin lesion categories in the dataset including macule, patch, papule, plaque, vesicle, bulla, pustule, nodule, atrophy, scaling, crust, tylosis, and excoriation classes.

## 4 EXPERIMENTAL RESULTS

In this paper, we investigate the inference performance of Bayesian‐Edge Intelligence design, evaluating its prediction accuracy and convergence performance. We also compare the prediction performance of our proposed model with that of the state‐of‐the‐art (non‐Bayesian models used in other studies for the classification and segmentation tasks of skin lesions. Then, we analyze the obtained model uncertainty to see if it helps rank the sample predictions, referring them for further inspection and correction and improving the overall model performance. We finally shed light on the Bayesian‐Edge model to find the underlying causes of model performance. We analyze distinct probabilistic versions of the VGG‐16, ResNet‐50, and DenseNet‐169 architectures to the criteria to find the approximate Bayesian variants with the prediction performance. Table 2 summarizes our implemented model's prediction accuracy and state‐of‐the‐art models proposed in other studies, as shown in Figure 6.

**TABLE 2:** Quantitative comparison of the implemented models in skin lesion classification and segmentation of HAM dataset.

Skin lesion models	Classification and segmentation accuracy
VGG‐16	81.50
ResNet‐50	80.04
Denssenet‐121	82.70
Bayesian‐Edge model	87.80

**FIGURE 6:** Quantitative comparison of skin lesion classification and segmentation models.

According to the data in the table about different models, the Bayesian‐Edge model significantly outperforms the rest. It also performs on par with or marginally better than the state‐of‐the‐art models, except some of the models presented, which exploit additional auxiliary processing stages to improve the performance, such as working with crops of the high‐resolution images instead of down‐sampling conducting an extensive multi‐crop evaluation, employing an ensemble of CNNs and a meta‐learning step via training an auxiliary SVM classifier. However, our proposed Bayesian‐Edge model can detect and classify the images of skin lesions more accurately.

RETRACTED

## 5 RESULTS AND DISCUSSION

This study introduces two distinct methodologies, Bayesian Inference and Edge Intelligence, for segregating skin lesions. Multiple instances of Bayesian Inference have been examined, and an approach for conducting skin detection using a combination of labeled and unlabeled data are proposed. When confronted with employing labeled and unlabeled data for skin detection through Bayesian Inference, our analysis recommends adopting the subsequent approach: Initiate the process with Naïve Bayes, focusing on learning solely from the existing labeled data. Subsequently, validate the model's accuracy by refining it with unlabeled data.

If the outcomes are deemed satisfactory, the integration of edge intelligence can potentially be pursued to enhance performance. Should none of the techniques involving unlabeled data yield performance improvements beyond supervised learning (Naïve Bayes), practitioners encounter two alternatives: disregard the unlabeled data or employ the active learning approach to label a subset of the unlabeled data. Naturally, active learning becomes feasible if the resources to label specific samples are available. The utilization of unlabeled data does not exclusively prompt the exploration of structure learning within Bayesian inference. It is important to note that the challenge of skin detection could be addressed using classifiers beyond Bayesian inference. However, such a solution would essentially comprise a fusion of three components:^37^

1. The idea demonstrates the drawbacks of using unlabeled data as motivation.
2. The creation of algorithms to look for Bayesian inference structures that perform better.
3. The successful use of labeled and unlabeled data learning for skin detection.

We have also examined the effectiveness of our various tactics in Table 3 and Figure 7. On the segmentation data, we mainly compare how Edge Intelligence and Bayesian Inference perform. Our segmentation algorithm's performance has been evaluated on a class‐by‐class basis.

**TABLE 3:** Comparison between Bayesian inference and edge intelligence.

Model	DI	JI
Edge intelligence	0.813	0.734
Bayesian inference	0.852	0.767

Abbreviations: DI, dice coefficient; JI, Jaccard index.

**FIGURE 7:** Comparison between Bayesian inference and edge intelligence.

Skin lesions are an essential health issue. Various techniques are applied to segment the skin lesions infected data from images. This research paper presents a skin lesion segmentation approach based on the elitist‐Java Optimization algorithm and Bayesian Inference approach. These approaches consist of two metrics: The dice coefficient (DI) and the Jaccard index (JI). The experimental samples comprised 320 images from the skin lesion datasets. These performance metrics, namely accuracy, DI, senility, and specificity, are applied to evaluate the execution of the segmentation approach and the computation time. The outcomes proved that the proposed approach improved the segmentation accuracy of the affected skin lesions area and outperformed the compared methods.

RETRACTED

As evident from the data presented in Table 3, Bayesian Inference notably surpasses Edge Intelligence in terms of performance on the test data. This discrepancy could be attributed to the Bayesian Inference's capacity to detect the edges of skin lesions effectively. The incorporation of Edge Intelligence, however, contributes to an overall enhancement of our proposed system's performance. The Bayesian inference framework yields posterior probability distributions encompassing the seven distinct classes. The assembled dataset was employed throughout the experimental process, with the segregation model being trained and tested on a total of 10 000 images. The K‐fold cross‐validation strategy was adopted for training and testing the segregation model. The dataset is partitioned into K equal subsets in this technique, and a holdout procedure is iterated K times. During each iteration, the Kth subset is utilized for testing, while the remaining K‐1 subsets are used for training. Ultimately, the average performance is computed across all K trials. Leveraging a comprehensive set of 35 color and texture features, Edge Intelligence is the most effective classifier among all alternatives.^38^

In Table 4 and Figure 8, the performance of different classifiers is elaborated upon the 10‐fold cross‐validation outcomes. The values represent mean scores along with their corresponding standard deviations. The values highlighted in bold indicate the most optimal accuracy, sensitivity, and specificity scores. A system for improving asymmetry classification in the PH2 dataset using dermatologist‐like feature extraction from skin lesions is discussed in Chakravorty et al.^39^ Early diagnosis of melanoma was performed using asymmetry according to medical algorithms such as ABCD and CASH. They presented the performance of several classifiers using these features. The obtained result shows better asymmetry classification than the available literature. The results for complete asymmetry using SVM were accuracy (81.74%), sensitivity (82.01%), and specificity (87%).  To enhances the performance of multi‐class skin classification is discussed in Debelee.^40^ An Edge intelligence technique was developed to lessen the effects of the major‐type misclassification issue. The major‐type and multi‐class classification performances were balanced using the late fusion method. The dataset was used in a series of tests by the author to assess the performance of the suggested approach. The experimental results demonstrated that the proposed method outperformed the representative DP algorithms for skin lesion categorization in all assessment metrics in his study for accuracy, sensitivity, and specificity in the major‐type categorization. Edge intelligence scored 87.80%, 84.38%, and 88.68%, respectively. Regarding the sensitivity of the minority classes, Edge intelligence performed better than the Quadratic SVM model.  Aryan et al. Bayesian inference can improve the performance of the machine‐physician team in the skin lesion classification task.^41^ They used the skin lesion dataset, which includes samples from seven common skin lesion categories shown in Figure 2. They show that Bayesian inference can boost diagnostic performance by 88.16%, 86.48%, and 90%, respectively, without incurring additional parameters or heavy computation. Moreover, the Bayesian inference technique reaches a classification accuracy of 90% while only referring 35% of the cases to physicians. The findings are expected to be generalized to other medical diagnosis applications. The availability of classification and segmentation methods will enable a wider adoption of ML technology in clinical settings.^42^, ^43^, ^44^, ^45^

**TABLE 4:** Comparison between different classifiers.

Classifier	Accuracy (SD)	Sensitivity (SD)	Specificity (SD)
Quadratic SVM	81.74%	82.01%	87.00%
Edge intelligence	87.80%	84.38%	88.68%
Bayesian inference	90.00%	86.48%	88.80%

RETRACTED

**FIGURE 8:** Comparison between different clusters.

## 6 CONCLUSION

In this study, we present a Bayesian‐Edge model, which outputs an estimate of the model accuracy with no additional parameter or significant change in the architecture for detecting and classifying skin lesion images. Our proposed model makes a prediction only when it is highly confident about its competency and refers the case to physicians. Our experimental results in the skin lesion classification images show that the Bayesian‐Edge model achieves a higher prediction diagnosis than the state‐of‐the‐art models. We show that imposing approximate Bayesian inference increases the diagnosis performance by 88.80%. Moreover, the prediction accuracy reaches nearly 90% on the remaining samples when exploiting the model accuracy to refer, respectively, 25% and 40% of the most uncertain samples for further examination. This property enables a hybrid physician model that saves human effort while maintaining high diagnostic accuracy. The proposed mechanism is general and applicable to any medical image classification task involving skin lesion images, the image's edge, and the images' effectiveness. In the future, this technology will enable broader adoption in clinical settings to investigate the possibility of sending the estimates of the image's accuracy as feedback information to modify and improve its prediction capability directly. In addition, the researchers may also focus on incorporating advanced hybrid machine learning and blockchain‐based mechanisms^46^, ^47^, ^48^, ^49^, ^50^ to enhance data security.

RETRACTED

## CONFLICT OF INTEREST STATEMENT

The authors declare no conflicts of interest.

## Data Availability

The data will be available upon reasonable request to the corresponding author.
